The article "Data Confidentiality in Healthcare Monitoring Systems Based on Image Steganography to Improve the Exchange of Patient Information Using the Internet of Things" was published in 2022. Journal: J Healthc Eng.

# Data Confidentiality in Healthcare Monitoring Systems Based on Image Steganography to Improve the Exchange of Patient Information Using the Internet of Things

**DOI:** 10.1155/2022/7528583

**Published:** 2022-05-06

**Authors:** Hussah N. AlEisa

**Affiliations:** Department of Computer Sciences, College of Computer and Information Sciences, Princess Nourah Bint Abdulrahman University, Riyadh 11671, Saudi Arabia

## Abstract

Recently, with the availability of fast and reliable Internet, the distance between a patient and a doctor is becoming unimportant. Physicians will be able to request the medical images of their patients regardless of the geographical area. However, a lot of challenges face such successful implementation. To facilitate remote diagnosis, patient electronic medical record (EMR), including medical images, that originates in one system needs to be exchanged either within the same organization or across different organizations. Steganography is the practice of concealing a secret message inside a cover medium. In this paper, steganography will be used to embed the patient's personal information securely and imperceptibly in their medical images to enhance confidentiality in case of a distant diagnosis. The security of the medical data is improved to maintain confidentiality and integrity using IoT. The least significant bit of the approximate coefficient of integer wavelet transform is proposed. The distortion between the cover image and stego-image is obtained by measuring the mean square error and PSNR, and normalized cross-correlation is utilized to estimate the degree of closeness between the cover image and stego-image.

## 1. Introduction

Communication through digitized media has been increasingly evident with the development of the Internet. All individual and commercial communication takes place on the Internet, where computerized media is the primary means. When sensitive data from businesses and organizations is shared, the security of the information is a major problem. They are required to keep their data safe from interfering eyes. However, everyone in today's world has access to the Internet, so there is a great danger in transmitting data digitally. The conservation of data during transmission is addressed in this way [1].

In today's world, the confidentiality of secret data is paramount, and advances in the security of computers have positioned steganography as a superior technique for acquiring secured data. Steganography is the method of concealing secret data in a message, audio file, picture, or video by embedding it in another image, audio file, video, or message [2–4]. It is used to keep sensitive information safe from hackers. Nowadays, the volume of data shared via the Internet is expanding. As a result, data security is considered a severe concern when data is communicated through the Internet [5, 6].

The article "Data Confidentiality in Healthcare Monitoring Systems Based on Image Steganography to Improve the Exchange of Patient Information Using the Internet of Things" was published in 2022. Journal: J Healthc Eng.

In steganography methods, each pixel of the cover picture is hidden with an equivalent number of secret bits. The embedding alteration in the cover image is equal. Individual pixels in a digital picture, on the other hand, have complicated statistical connections. As a result, the picture quality is automatically lowered while modifications with equal number of bits are made in the cover image pixel [7]. Different adaptive embedding techniques have been included within the steganography method to address these concerns. Each pixel of the cover picture is embedded with a changing number of bits using this adaptive embedding approach. As a result, the majority of researchers concentrated on adaptive strategies to increase the safety of the steganography approach [8–12]. Additionally, the value of edge pixels is unaffected by modifications made during the embedding process. As a result, edge pixels can hold more hidden bits than smooth pixels. In most applications, metaheuristic algorithms are employed to tackle optimization problems [13–16].

To safeguard data, IoT transmitted data in the cloud through the Internet is employed. High data security is provided via complicated encryption and decryption technology. Only encryption and decryption are used, but data concealment offers a greater benefit [17, 18].

For security difficulties in the data communication between two devices in an IoT network as shown in Figure 1, several security criteria such as authentication, integrity, and secrecy were applied. Attacks are classified as low-, medium-, high-, and extremely high-level attacks based on their behavior and threat level.

The two types of image steganographic methods are spatial domain and frequency domain [19]. Spatial domain approaches deal with the direct change of picture pixels, and while they have a higher payload and imperceptibility, they are vulnerable to statistical assaults [20]. Frequency domain approaches, on the other hand, use changed coefficients resulting from different transformations such as DWT, DFT, and DCT for data embedding. These approaches are more resistant to image processing assaults, but they are computationally demanding and have a small payload, making them unsuitable for real-time applications [21, 22].

There are two ways to classify steganography techniques. Steganography methods are classified into image steganography, video steganography, text steganography, audio steganography, and network steganography, depending on the kind of cover image [23]. Steganography techniques are divided into two categories based on the embedding domains: spatial domain techniques, such as least significant bit and pixel value differencing approaches; transform domain techniques, such as discrete cosine transform (DCT), discrete wavelet transform (DWT), and integer wavelet transform (IWT); spread spectrum systems; masking distortion systems; and filtering methods [24].

The article "Data Confidentiality in Healthcare Monitoring Systems Based on Image Steganography to Improve the Exchange of Patient Information Using the Internet of Things" was published in 2022. Journal: J Healthc Eng.

## 2. Related Work

For securing information in an IoT architecture, three-color picture steganography algorithms are proposed. The first and third techniques employ red, green, and blue components for information transmission, whereas the second technique utilizes green and blue components. The dynamic positioning techniques were developed by utilizing the shared secret key to hide data in the deeper layer of the image channels [25].

The performance analysis of the secret image steganography technique for the security of images and data is discussed. For image steganography, modified LSB replacement and data mapping algorithms have been developed. Initially, the secret picture was preprocessed utilizing the data mapping method which was used to embed the secret picture in the cover image. In general, the majority of LSB approaches did not rely on pixel correlation or picture content. As a result, it might be detected through RS analysis. Consequently, some preventive measures are required to enhance the security of LSB-based steganography approaches. An edge detection procedure has been implemented in the LSB-based steganography approach to address this problem. Furthermore, before incorporating the secret images into the cover image, they should be encrypted to increase security. Due to the lack of encryption methods preceding the embedding process, the security level of several current approaches has been decreased [26].

The data secured in the fog cloud IoT system is presented. The user in one region of the system uploads substantial data using the suggested quantum steganography convention and then transmits the protected data to the fog cloud. The intended receiver receives the data from the mist cloud and extracts the anticipated material using the specified extraction method [27].

A method for encrypting any form of an image, particularly medical images, has been developed. They intended to secure the integrity of electronic medical data while also sustaining its availability and authentication to ensure that only authorized personnel had access to it. In the first stage, the AES encryption technology was used. With seven values retrieved from the ear image as feature vectors, the ear print is also included. By delivering medical pictures over the Internet, the suggested approach increased the security of these images and protected them from unauthorized access [28].

The article "Data Confidentiality in Healthcare Monitoring Systems Based on Image Steganography to Improve the Exchange of Patient Information Using the Internet of Things" was published in 2022. Journal: J Healthc Eng.

The decision tree approach is used to present a novel method for shifting the medical data of the patient by securing the data into the medical cover image. The encryption is performed in the form of several chunks which are disseminated uniformly. Secret numbers are allocated to the cover image in the mapping method based on the breadth-first search to insert the data. Before embeddings, the data was encrypted using the RSA technique [29].

A safe approach that can meet the security and protection requirements while also overcoming the SPECS flaws is offered. In addition, this demonstrates the plan's success through execution assessments in terms of confirmation postponement and transmission overhead [30].

Developments and security adjustments attempting to solve the vulnerabilities of the security approach are presented to overcome the instinctive safety flaws of the 2-factor substantiation method. The proposed security enhancements may be used with the 2-factor authentication approach to achieve a more secure and robust two-factor client verification through WSNs [31]. For embedding reasons, the interblock approach is utilized. Images in the JPEG format are referred to as host or stego-images. This approach is only used to conceal patient information in medical JPEG photos. The difference in the coefficients is calculated using discrete cosine transform (DCT) [32].

In today's healthcare systems, Internet of Things (IoT) devices play a critical role. To incorporate patient data in any cover media, 2D DWT is applied. For the cover photos, grayscale and color photographs are utilized. Text data is encrypted using standard methods before being embedded in the cover medium. Various numerical methods are used to validate the imperceptibility of the cover image [33, 34].

On the segmented image, the region of the object and the reversible watermarking technique are employed. If image modes such as X-rays, magnetic resonance imaging (MRI), or computed tomography (CT) images have been tampered with or forged, the presented methodologies perform effectively to identify the tampering using the hash code. As medical systems are more prone to fabrication or manipulation, reversible watermarking methods are particularly useful [35, 36].

Steganography is a method for embedding data in many images, as compared to classical steganography, which uses just one image at a time for embedding. In the event of an exceptional state in the communication media during data transmission, secret data bits can be recovered from many shares. Compressed JPEG images are extensively useful for communication channels. An intermediate image is constructed before transmitting it to the channel, which is near enough to the stego-image [37].

The article "Data Confidentiality in Healthcare Monitoring Systems Based on Image Steganography to Improve the Exchange of Patient Information Using the Internet of Things" was published in 2022. Journal: J Healthc Eng.

A novel method for securing secret data in a fingerprint image created from a hidden message is proposed. Unlike traditional steganography techniques, there is no requirement for a cover signal for the embedding process. The secret message is transferred to the polynomial, encoded at diverse points of polarities, and utilized as a portion of the hologram to generate the fingerprint image [38–40].

## 3. Methodology

This section discusses the proposed methodology for maintaining data confidentiality during the IoT distribution process. Because information is passed across numerous hops in the Internet of Things, data security is critical. Due to the ease with which data may be accessed, the mixture of various gadgets and the interconnections established through a multitude of data give space for privacy breaches in IoT. As a result, in such a case, data may be secured by a reliable encoding technique. Accordingly, this study proposes a dependable data transmission model for a safe IoT connection, as shown in Figure 2, which is a depiction of a setup in healthcare that uses an IoT dispersed structure.

### 3.1. Steganography

A steganography approach based on encryption is proposed for conveying secret data. Normally, a digital image consists of disparate picture parts known as pixels. As a cover picture, a grayscale image and a color image are utilized in this work. As a result, a picture is represented by a large array of bytes. Image encryption, embedding phase, quality improvement, and extraction phase are the four key aspects of the system proposed. This programme is commonly used in photos, although the method's characteristics are generally stated in some figures, including hash marking. Steganography protects against unauthorized users and illegal copyrights.

Steganography is a progression in which secret data is hidden so that its presence cannot be recognized. This is why steganography is sometimes referred to as “covered writing.” The goal of steganography is not only to secure the encryption but also to hide it so that no one can detect or determine the presence of the hidden secret data. This system or technique aims to hide the presence of any secret data. The person who is not permitted to push for knowledge access should not even know if any secret information is available.

The basic components of steganography are the message, the carrier and the stego-key. The message is that the secret text, image, video, or audio has to be safeguarded using the steganography process. The carrier is the path or medium through which the key and, hence, the covered message are sent. The stego-key is the password by which confidential data is protected and exposed as shown in Figure 3.

The article "Data Confidentiality in Healthcare Monitoring Systems Based on Image Steganography to Improve the Exchange of Patient Information Using the Internet of Things" was published in 2022. Journal: J Healthc Eng.

### 3.2. Image Encryption

In the encryption process, the hidden image is processed with binary by plane decomposition which is utilized to decompose the image into binary bit planes. The image is represented with binary planes in this method for a decimal number which is given as

(1) $$\begin{array}{c} B=\sum_{i=0}^{n-1}b_{i}2^{i},\\ B=b_{0}2^{0}+b_{1}2^{1}+\cdots \cdots \cdots +b_{n-1}2^{n-1},\\ B=b_{0}+2b_{1}\cdots \cdots \cdots \cdots \cdots +2^{n-1}b_{n-1}. \end{array}$$

The grayscale image has the pixel value in the range of 0 to 255, which is decomposed into binary bit values. With the support of secret key binary, keystreams are generated. These binary keystreams enter the two stages of the encryption model. The piecewise linear chaotic map is utilized to produce the keystreams, which are represented as

(2) $$\begin{array}{c} x_{i+1}=\left\{\begin{array}{cc} \frac{x_{i}}{\delta }, & 0\leq x_{i}\leq \delta ,\\ \frac{x_{i}-\delta }{0.5-\delta }, & \delta \leq x_{i}\leq 0.5,\\ F\left(1-x_{i},\delta \right), & 0.5\leq \delta \leq 1. \end{array}\right. \end{array}$$

The control parameter is represented as *δ*, and *x*_*i*_ provides the initial condition of piecewise linear chaotic mapping. The set of the hidden image *δ* is encrypted with the initial value *x*_0_

The keystream *X*={*x*_1_, *x*_2_,……*x*_*n*_} is converted into the integer sequence *X*_1_(*i*).

(3) $$\begin{array}{c} X_{1}=\mathrm{mod}\left(\text{floor}\left(X\times 10^{14}\right),256\right). \end{array}$$

The bit-plane decomposition utilizes the keystream into bit planes to obtain the binary sequence *k*_1_ and *k*_2_ in which the bits are arranged from a higher bit plane to a lower bit plane.

#### 3.2.1. Diffusion Stage

The diffusion stage is performed by the following steps.

(1) Elements *M* are added as
  (4) $$\begin{array}{c} S_{1}=\sum_{i-0}^{n-1}M_{1}\left(i\right). \end{array}$$
(2) Cyclic operation is performed in *M*_1_ to obtain the matrix *M*_11_, and *M*_1_ element is shifted right by *S*_1_ bits.
(3) First element *M*_1_ is encrypted, and the key of the first element *M*_1_ is given as
  (5) $$\begin{array}{c} P_{1}\left(i\right)=M_{11}\left(i\right)⊕M_{11}\left(i-1\right)⊕M_{2}\left(i\right)⊕k_{1}\left(i\right). \end{array}$$
(4) Element P is given as
  (6) $$\begin{array}{c} S_{2}=\sum_{i=1}^{n-1}P_{1}\left(i\right). \end{array}$$
(5) Cyclic operation is performed in *M*_2_ to obtain the matrix *M*_22_, and *M*_2_ element is shifted right by *S*_2_ bits.
(6) First element *M*_22_ is encrypted, and the key of the first element *M*_2_ is given as
  (7) $$\begin{array}{c} P_{2}\left(i\right)=M_{22}\left(i\right)⊕M_{22}\left(i-1\right)⊕P_{1}\left(i\right)⊕k_{1}\left(i\right). \end{array}$$

The article "Data Confidentiality in Healthcare Monitoring Systems Based on Image Steganography to Improve the Exchange of Patient Information Using the Internet of Things" was published in 2022. Journal: J Healthc Eng.

#### 3.2.2. Confusion Stage

The steps performed in confusion matrix are given as follows.

(1) The elements *P*_1_ and *P*_1_ are added as given below:
  (8) $$\begin{array}{c} S_{3}=\sum_{i=0}^{nm}P_{1}\left(i\right)+P_{2}\left(i\right). \end{array}$$
(2) The keystreams *k*_1_ and *k*_2_ are generated using the secret key *k*(*x*, *δ*). The initial value *a*_0_ is generated using the following:
  (9) $$\begin{array}{c} a_{0}=\mathrm{mod}\left(\frac{a_{0}+S_{3}}{nm,1}\right). \end{array}$$
(3) The chaotic sequence is generated as
  (10) $$\begin{array}{c} A_{1}=\left\{a_{1},a_{2},\ldots \ldots \ldots .a_{nm}\right\},\\ A_{2}=\left\{a_{nm+1},a_{nn+2},\ldots \ldots \ldots .a_{nm}\right\}. \end{array}$$
(4) The integer sequence *X*_1_ and *X*_2_ is given as
  (11) $$\begin{array}{c} X_{1}=\mathrm{mod}\left(\text{floor}\left(A_{1}\times 10^{14}\right),4nm\right)+1,\\ X_{2}=\mathrm{mod}\left(\text{floor}\left(A_{2}\times 10^{14}\right),4nm\right)+1. \end{array}$$
(5) The row vector *R*_1_ is obtained by encrypting the swapping elements *P*_1_ and *P*_2_:
  (12) $$\begin{array}{c} \text{temp}=P_{1}\left(i\right),\\ P_{1}\left(i\right)=P_{2}\left(X_{1}\left(i\right)\right),\\ P_{2}\left(X_{1}\left(i\right)\right)=\text{temp.} \end{array}$$
(6) The row vector *R*_2_ is obtained by encrypting the swapping elements *P*_1_ and *P*_2_:
  (13) $$\begin{array}{c} \text{temp}=P_{2}\left(i\right),\\ P_{2}\left(i\right)=P_{1}\left(X_{2}\left(i\right)\right),\\ P_{1}\left(X_{2}\left(i\right)\right)=\text{temp.} \end{array}$$
(7) *R*_1_ and *R*_2_ are the row vectors which are transformed into *n*×*m* images to obtain the secret image.

### 3.3. Embedding Process

The embedding approach involves some cover image and secret image preparation, as well as secret key extraction and data hiding. The cover picture was chosen based on certain conclusions drawn from earlier steganography studies. This should be done carefully so that the superiority of the stego-image created after hiding is preserved. Certain pixels or blocks are chosen from the cover image using a random key. Before embedding, the secret picture is compressed and encrypted. Compression reduces the quantity of data to be hidden, while encryption improves security. Even if the primary concern of steganography is exploited, data should not be exposed. The secret image is compressed using a sophisticated wavelet-based compression algorithm. Simple bit operations like AND and OR are used to encrypt data. After that, the secret picture is transformed into a bitstream, referred to as the secret data. The LSB approach is utilized to disguise the secret data in the chosen pixels. It is sufficient to swap the final two bits if the quantity of data is less. Otherwise, the secret data is swapped for the least significant 3 bits of the chosen pixels to generate the stego-image as shown in Figure 4.

The article "Data Confidentiality in Healthcare Monitoring Systems Based on Image Steganography to Improve the Exchange of Patient Information Using the Internet of Things" was published in 2022. Journal: J Healthc Eng.

### 3.4. LSB Domain Algorithm

The algorithm for hiding a hidden text in an image is the LSB. The LSB embedding technique uses the secret text bitstream to be hidden to substitute the LSBs of the pixels in the cover picture. Because deviations in the LSBs of pixels do not produce variation in the image, the stego-image is virtually identical to the cover image.

The pixel value *I*(*a*, *b*) of LSB is similar to message bit which is embedded in *I*(*a*, *b*), and it remains unchanged. The stego-image is obtained as follows:

(14) $$\begin{array}{c} I_{s}\left(a,b\right)=\left\{\begin{array}{cc} I\left(a,b\right)-1, & m=0,\text{LSB}\left(I\left(a,b\right)\right)=1,\\ I\left(a,b\right), & \text{LSB}\left(I\left(a,b\right)\right)=m,\\ I\left(a,b\right)+1, & m=0,\text{LSB}\left(I\left(a,b\right)\right)=1\text{,} \end{array}\right. \end{array}$$

where *m* is the next bit for embedding each pixel by changing a bit.

The pixels of an image must be adjusted to incorporate a hidden message. It is hard to differentiate between the cover image and the stego-image. This approach often generates significant distortion in the cover image when the number of hidden bits for each pixel reaches three. There are many steganographic to be utilized to mitigate the distortion induced by LSB replacement. Adaptive approaches alter the number of concealed bits in each pixel, resulting in a higher image quality compared to systems that rely only on LSB replacement. However, this comes at the expense of lowering the embedding capacity.

### 3.5. IWT Technique

An integer data set is transformed into another integer data set using the IWT. When the data is hidden in the coefficients of the wavelet filters used in the DWT, any method that is most effective for the floating-point values of the pixels that should be integers may result in the loss of the hidden data, failing the data hiding system. To avoid difficulties with wavelet filters' floating-point accuracy when the input data is an integer, such as in digital images, the output data will no longer be an integer, preventing perfect recreation of the original image and preventing information loss through forward and inverse transforms. The lifting technique is one of the approaches for performing the IWT. IWT can transform integer wavelet coefficients from pixel values and recreate the image from integer wavelet coefficients due to its numerical advantages.

The article "Data Confidentiality in Healthcare Monitoring Systems Based on Image Steganography to Improve the Exchange of Patient Information Using the Internet of Things" was published in 2022. Journal: J Healthc Eng.

The image pixel is decomposed into four subband wavelets of DWT: LL, LH, HL, and HH. The coefficient of the image is approximated using the LL subband, vertical details of the image are given using the LH subband, horizontal details of the image are examined in HL, and diagonal details of the image are given using the HH subband. The coefficient of IWT is computed as

(15) $$\begin{array}{c} LL_{a,b}=\left[\frac{\left(I_{2a,2b}+I_{2a,2b}\right)}{2}\right],\\ LH_{a,b}=I_{2a,2b+1}-I_{2a,2b},\\ HL_{a,b}=I_{2a+1,2b}-I_{2a,2b},\\ HH_{a,b}=I_{2a+1,2b+1}-I_{2a,2b}. \end{array}$$

The coefficient of inverse IWT is given as

(16) $$\begin{array}{c} I_{2a,2b}=LL_{a,b}-\left[\frac{HL_{a,b}}{2}\right],\\ I_{2a,2b+1}=LL_{a,b}-\left[\frac{HL_{a,b+1}}{2}\right],\\ I_{2a+1,2b}=I_{2a,2b+1}+LH_{a,b}-HL_{a,b},\\ I_{2a+1,2b+1}=I_{2a+1,2b}+HH_{a,b}+LH_{a,b}. \end{array}$$

The steps of the algorithm for the embedding process in IWT-LSB are as follows:

1. The cover image is read.
2. The secret image is read.
3. IWT is applied for the cover image.
4. Change the LSB of the coefficient image by the secret image.
5. Until the secret data is completely hidden in the cover image, step 4 will be continued.
6. Inverse IWT is applied.
7. Stego-image is obtained.

### 3.6. Image Quality Enhancement

The obtained stego-image from the embedding process is of insufficient quality. As a result, a processing procedure on the unique intelligent system is required. This phase is necessary for reducing the chances of numerical identification and other types of image modification attempts.

### 3.7. Hybrid Fuzzy Neural Network

An HFNN with a backpropagation learning method is employed to improve the image quality in this study. In general, neural networks resemble HFNNs that are inhomogeneous. The neural network refers to a framework that can simulate how the human brain learns. The stego-image transformed to binary bit values in order to identify free bits and bits that encompass secret bits. A buffer is built to keep the free bits that are not used by the embedding process. The stego-and cover images are also used to extract statistical and perceptual attributes. The statistical and visual aspects are represented by the chi-square probability and the Euclidian norm. The HFNN is provided with the free bits buffer as well as the two characteristics of the stego-image. The cover attributes are then compared to the HFNN outputs. By integrating the changed free bits with the secret bits, a new stego-image is created if the outputs match the characteristics of the cover image. The HFNN weights are modified using a backpropagation learning process.

1. The stego-image is generated by hiding the secret image, which is implemented using embedding approach algorithms.
2. Features are extracted from the stego-image using the feature extraction technique.
3. A buffer is generated which is not utilized in the steganographic algorithm. The secret is not hidden in the buffer bit, and it is called free bits.
4. The statistical and visual measure of the stego-image is measured using a fuzzy neural network with backpropagation. The statistical and visual measure of the stego-image is measured using a fuzzy neural network with backpropagation. Therefore, for an updated stego-image, the free bit buffer, statistical and visual measures are contained in the output layer.
5. The output of the fuzzy network is compared with the cover image. The stego-image is formed if the output and cover image get matched and the output with the free bit is used by assembling the other bit in which the secret image is hidden. Otherwise, step 4 is repeated.

The article "Data Confidentiality in Healthcare Monitoring Systems Based on Image Steganography to Improve the Exchange of Patient Information Using the Internet of Things" was published in 2022. Journal: J Healthc Eng.

The input layer, rule layer, fuzzification layer, inference layer, and defuzzification layer are the five layers that compose HFNN as shown in Figure 5. The input neurons of the HFNN were trained using five layers of backpropagation, using inputs from the free bits buffer, and numerical and graphic characteristics. Following that, all hidden neurons in the fuzzification layer get the inputs. The membership function is used to perform fuzzy process on input characteristics at this layer. For the excellent approximation of input space, the Gaussian membership function is utilized. By altering the parameter values, this bell-shaped function produces several membership functions for the input characteristics. The strength of fuzzy rules is determined in the rule layer using the logical AND operator. On fuzzy inference, the inference layer executes OR operations. The HFNN output will emerge from the defuzzification layer. The weight parameter is used to link the nodes of all layers in HFNN.

The dimensionality reduction is a feature extraction in which set of features is transformed form stego image. The statistical features are obtained from chi-square probability and visual features from the Euclidean norm. Let *x* and *y* be the input, then linguistic input variable *A*_1_, *A*_1_ and *B*_1_, *B*_1_. The linguist state is given as

(17) $$\begin{array}{c} A_{j}\left(u\right)=\exp\left[-\frac{1}{2}{\left(\frac{a-u_{j1}}{v_{j1}}\right)}^{2}\right],\\ B_{j}\left(u\right)=\exp\left[-\frac{1}{2}{\left(\frac{a-u_{j2}}{v_{j2}}\right)}^{2}\right]. \end{array}$$

{*u*_*j*1_, *u*_*j*1_, *u*_*j*1_, *u*_*j*1_} are the parameter set. The logical operator is used to strength the output of the network layer:

(18) $$\begin{array}{c} F_{1}=A_{1}\left(x_{0}\right)\Lambda B_{1}\left(y_{0}\right),\\ F_{2}=A_{2}\left(x_{0}\right)\Lambda B_{2}\left(y_{0}\right). \end{array}$$

The defuzzification is obtained as the normalization:

(19) $$\begin{array}{c} F_{d1}=\frac{F_{1}}{F_{1}+F_{2}},\\ F_{d2}=\frac{F_{2}}{F_{1}+F_{2}}. \end{array}$$

The error function is given by

(20) $$\begin{array}{c} E=\frac{1}{2}{\left(y-0\right)}^{2}. \end{array}$$

The desired output is represented as *y*.

The article "Data Confidentiality in Healthcare Monitoring Systems Based on Image Steganography to Improve the Exchange of Patient Information Using the Internet of Things" was published in 2022. Journal: J Healthc Eng.

### 3.8. Extraction Process

The extraction process is used to extract the hidden image from the embedded process in adjustable order. The cover image used in the first step is not used to extract the secret image. The data is provided by the LSB, and the procedure was enhanced using the secret key.

#### 3.8.1. Algorithm for Extraction Process in IWT-LSB

1. Stego-image is read.
2. Median filter is applied.
3. IWT is applied for stego-image.
4. The secret data is extracted for the approximate image coefficient of stego-image.
5. Until the secret data is extracted, step 4 will be continued.
6. Inverse IWT is applied.
7. Image gets extracted.
8. Extract the secret data.

### 3.9. Special Cases

#### 3.9.1. IWT-LSB Algorithm for Grayscale Image

The proposed hybrid IWT-LSB technique for grayscale images involves an embedding phase and an extraction phase as shown in Figure 6. In the embedding phase, the grayscale cover image is transformed using IWT, then the secret text is embedded in the LSBs of the cover image's coefficients, and finally the inverse IWT is used to construct the stego-image. Without knowing anything about the original image, the hidden text might be extracted throughout the extraction process. The hidden secret text is retrieved from the LSBs of the filtered stego-image's coefficients, and the inverse IWT is useful for creating the extracted image.

The 512 × 512 bitmap grayscale images are utilized as cover images for the hybrid IWT-LSB algorithms on grayscale images. The size of the estimated coefficient images after performing the IWT is 256 × 256, which implies that a secret text with up to 8 and 192 digits may be secured. To improve the system's robustness and secure the message from external impacts such as noise, compression, and filtering, the secret data is placed in the LSBs of the estimated coefficient images of the cover images.

#### 3.9.2. IWT- LSB Algorithm for Color Image

The color image is split into R, G, and B components in the proposed methodology, and the three components are employed to hide data as shown in Figure 7. In the embedding phase, the RBG component is used to decompose the color of cover image in which the IWT transform is used with the signature of the user and the secret data is embedded with actual length in LSB and coefficient image is approximated for the red component of cover image. The image's approximated green and blue components coefficient are used to secure the secret data. Then, the inverse IWT is applied to each component once the embedding process is complete, and then these components are recombined to generate a stego-image.

The article "Data Confidentiality in Healthcare Monitoring Systems Based on Image Steganography to Improve the Exchange of Patient Information Using the Internet of Things" was published in 2022. Journal: J Healthc Eng.

The hidden data may be extracted during the extraction process without knowing anything about the original image. The R, G, and B components are decomposed from the noisy stego-image in which median filter is utilized for filtering and then transformed using IWT. The LSB of the approximated image coefficient is used for extracting the actual length of the secret image by utilizing the G and B components, and the inverse IWT is utilized to extract the original image.

## 4. Result and Discussion

The result of the IWT-LSB algorithm for the steganography image such as grayscale image and color image is analyzed. Parameters such as MSE, NCC, and PSNR are used for the performance evaluation. The error among the cover image and stego-image is examined using MES and PSNR and compared with the existing techniques.

The cover image is represented as *I*_*C*_, and stego-image is represented as *I*_*S*_. The mean square error is calculated using the following equation:

(21) $$\begin{array}{c} \text{MSE}=\frac{1}{nm}\sum_{a=0}^{m-1}\sum_{b}^{n-1}{\left[I_{S}\left(a,b\right)-I_{C}\left(a,b\right)\right]}^{2}. \end{array}$$

The peak to signal noise ratio is given as

(22) $$\begin{array}{c} \text{PSNR}=10\;\log\left(\frac{I_{\max}^{2}}{\text{MSE}}\right). \end{array}$$

The number of rows and columns is represented as *n* and *m*, and *I*_max_ is the maximum hold of the original image.

The similarity and dynamic extent of the cover image and secret image are quantified using the mean square error. The mean square error in the total number of pixels in color and grayscale image is given in Figure 8.

The PSNR of the suggested algorithm compared with the existing technique is given in Figure 9. The PSNR regulates the difference in the dynamic range of invisibility in cover image and secret image in which the value is greater than 53 dB in grayscale and color image compared to the existing techniques.

The degree of closeness between the cover image and stego-image is obtained using NCC which is shown in Figure 10. The degree of closeness is obtained after embedding the data in the secret image.

The article "Data Confidentiality in Healthcare Monitoring Systems Based on Image Steganography to Improve the Exchange of Patient Information Using the Internet of Things" was published in 2022. Journal: J Healthc Eng.

## 5. Conclusion

This paper used image steganography to securely and imperceptibly embed the patient's personal information in their medical images to enhance confidentiality in case of distant diagnosis. The least significant bit of the approximate coefficient of integer wavelet transform is proposed. This technique is analyzed for grayscale image and color image. IWT is utilized to hide the secret image in LSB in the grayscale image, while IWT with R, B, and G component is used for hiding the secret image in color image. The distortion between the cover image and stego-image is obtained by measuring the mean square error and PSNR, and the degree of closeness between the cover image and stego-image is estimated by utilizing the normalized cross-correlation. The result shows that the IWT-LSB technique can hide secret data with large length with better MSE, PSNR, and NCC.

## Figures and Tables

**Figure 1:** Data hiding and extraction for broadcasting between IoT devices.

**Figure 2:** Block diagram of the proposed methodology.

**Figure 3:** Steganography scheme.

**Figure 4:** Flowchart of the LSB-IWT embedding process.

**Figure 5:** Quality enhancement of stego-image using HFNN.

**Figure 6:** Proposed embedding and extraction process for grayscale image steganography.

**Figure 7:** Proposed embedding and extraction process for color image steganography.

**Figure 8:** Comparison of mean square in color and grayscale image using proposed and existing technique.

**Figure 9:** Comparison of PSNR in color and grayscale image using proposed and existing technique.

**Figure 10:** Comparison of NCC in color and grayscale image using proposed and existing technique.

## Data Availability

The data used to support the findings of this study are included within the article.

## References

[1] Altaay A. A. J., Sahib S. B., Zamani M. An introduction to image steganography techniques.

[2] Al-Afandy K. A., Faragallah O. S., ELmhalawy A., El-Rabaie E.-S. M., El-Banby G. M. High security data hiding using image cropping and LSB least significant bit steganography.

[3] Elhadad A., Hamad S., Khalifa A., Ghareeb A. (2017). High capacity information hiding for privacy protection in digital video files. *Neural Computing & Applications*.

[4] Hamad S., Khalifa A., Elhadad A. (2014). A blind high-capacity wavelet-based steganography technique for hiding images into other images. *Advances in Electrical and Computer Engineering*.

[5] Hashim M., Rahim M. (2017). Image steganography based on odd/even pixels distribution scheme and two parameters random function. *Journal of Theoretical and Applied Information Technology*.

[6] Krishna B. M., Santhosh C., Suman S., Shireen S. K. (2022). Systems, and computers, “evolvable hardware-based data security system using image steganography through dynamic partial reconfiguration. *Journal of Circuits, Systems, and Computers*.

The article "Data Confidentiality in Healthcare Monitoring Systems Based on Image Steganography to Improve the Exchange of Patient Information Using the Internet of Things" was published in 2022. Journal: J Healthc Eng.

[7] Qin C., Zhang W., Cao F., Zhang X., Chang C.-C. (2018). Separable reversible data hiding in encrypted images via adaptive embedding strategy with block selection. *Signal Processing*.

[8] Li Q., Liao X., Chen G., Ding L. A novel game-theoretic model for content-adaptive image steganography.

[9] Khadse D. B., Swain G. (2021). Data hiding using quotient value differencing and remainder value substitution avoiding incorrect extraction problem. *Sensing and Imaging*.

[10] Sonar R., Swain G. (2022). A hybrid steganography technique based on RR, AQVD, and QVC. *Information Security Journal: A Global Perspective*.

[11] Sonar R., Swain G. (2021). Steganography based on quotient value differencing and pixel value correlation. *CAAI Transactions on Intelligence Technology*.

[12] Swain G., Pradhan A. (2022). Image steganography using remainder replacement, adaptive QVD and QVC. *Wireless Personal Communications*.

[13] Nipanikar S. I., Hima Deepthi V., Kulkarni N. (2018). A sparse representation based image steganography using particle swarm optimization and wavelet transform. *Alexandria Engineering Journal*.

[14] Swain G. (2018). Adaptive and non-adaptive PVD steganography using overlapped pixel blocks. *Arabian Journal for Science and Engineering*.

[15] Swain G. (2018). A data hiding technique by mixing MFPVD and LSB substitution in a pixel. *Information Technology and Control*.

[16] Swain G. (2019). Two new steganography techniques based on quotient value differencing with addition-subtraction logic and PVD with modulus function. *Optik*.

[17] Arunkumar S., Subramaniyaswamy V., Vijayakumar V., Chilamkurti N., Logesh R. (2019). SVD-based robust image steganographic scheme using RIWT and DCT for secure transmission of medical images. *Measurement*.

[18] Hureib E. S. B., Gutub A. A. (2020). Enhancing medical data security via combining elliptic curve cryptography with 1-LSB and 2-LSB image steganography. *International J Comp Sci Network Security (IJCSNS)*.

[19] Anees A., Siddiqui A. M., Ahmed J., Hussain I. (2014). A technique for digital steganography using chaotic maps. *Nonlinear Dynamics*.

[20] Xia Z., Wang X., Sun X., Liu Q., Xiong N. (2016). Steganalysis of LSB matching using differences between nonadjacent pixels. *Multimedia Tools and Applications*.

[21] Sajjad M., Muhammad K., Baik S. W. (2017). Mobile-cloud assisted framework for selective encryption of medical images with steganography for resource-constrained devices. *Multimedia Tools and Applications*.

The article "Data Confidentiality in Healthcare Monitoring Systems Based on Image Steganography to Improve the Exchange of Patient Information Using the Internet of Things" was published in 2022. Journal: J Healthc Eng.

[22] Elhadad A., Ghareeb A., Abbas S. (2021). A blind and high-capacity data hiding of DICOM medical images based on fuzzification concepts. *Alexandria Engineering Journal*.

[23] Kaur S., Bansal S., Bansal R. K. Steganography and classification of image steganography techniques.

[24] Thanikaiselvan V., Arulmozhivarman P. High security image steganography using IWT and graph theory.

[25] Abdelaziz A., Elhoseny M., Salama A. S., Riad A. M. (2018). A machine learning model for improving healthcare services on cloud computing environment. *Measurement*.

[26] Arya A., Soni S. (2018). Performance evaluation of secrete image steganography techniques using least significant bit (LSB) method. *International Journal of Computer Science Trends and Technology*.

[27] El-Latif A. A. A., Abd-El-Atty B., Hossain M. S., Elmougy S., Ghoneim A. (2018). Secure quantum steganography protocol for fog cloud internet of things. *IEEE Access*.

[28] Anwar A. S., Ghany K. K. A., Mahdy H. E. (2015). Improving the security of images transmission. *International Journal of Bio-Medical Informatics and E-Health*.

[29] Jain M., Choudhary R. C., Kumar A. Secure medical image steganography with RSA cryptography using decision tree.

[30] Horng S.-J., Tzeng S.-F., Pan Y. (2013). b-SPECS+: batch verification for secure pseudonymous authentication in VANET. *IEEE Transactions on Information Forensics and Security*.

[31] Khan M. K., Alghathbar K. (2010). Cryptanalysis and security improvements of ‘two-factor user authentication in wireless sensor networks’. *Sensors*.

[32] Liao X., Yin J., Guo S., Li X., Sangaiah A. K. (2018). Medical JPEG image steganography based on preserving inter-block dependencies. *Computers & Electrical Engineering*.

[33] Elhoseny M., Ramirez-Gonzalez G., Abu-Elnasr O. M., Shawkat S. A., Arunkumar N., Farouk A. (2018). Secure medical data transmission model for IoT-based healthcare systems. *IEEE Access*.

[34] Rostam H. E., Motameni H., Enayatifar R. (2022). Privacy-preserving in the Internet of Things based on steganography and chaotic functions. *Optik*.

[35] Eswaraiah R., Sreenivasa Reddy E. (2015). Robust medical image watermarking technique for accurate detection of tampers inside region of interest and recovering original region of interest. *IET Image Processing*.

[36] Sahu N., Peng D., Sharif H. (2021). Diagnosis-steganography-transmission: an innovative integrated paradigm for ECG healthcare. *SN Computer Science*.

[37] Al-Refai S., Al-Jarrah M. M. Secure data hiding technique using batch video steganography.

[38] Li S., Zhang X. (2018). Toward construction-based data hiding: from secrets to fingerprint images. *IEEE Transactions on Image Processing*.

The article "Data Confidentiality in Healthcare Monitoring Systems Based on Image Steganography to Improve the Exchange of Patient Information Using the Internet of Things" was published in 2022. Journal: J Healthc Eng.

[39] Taloba A. I., Sewisy A. A., Dawood Y. A. Accuracy enhancement scaling factor of Viola-Jones using genetic algorithms.

[40] Taloba A. I., Ismail S. S. An intelligent hybrid technique of decision tree and genetic algorithm for e-mail spam detection.

